The article "Diabetes regulated anti-inflammatory lncRNA is overexpressed in triple-negative breast cancer and predicts chemoresistance and tumor recurrence" was retracted in 2026. Reasons: concerns about the data; concerns about the results or conclusions.

# Diabetes regulated anti-inflammatory lncRNA is overexpressed in triple-negative breast cancer and predicts chemoresistance and tumor recurrence

**DOI:** 10.1080/21655979.2022.2068821

**Published:** 2022-05-24

**Authors:** Peng Wang, Wei Peng, Jian Peng

**Affiliations:** a Department of Physical Examination Center, Peking University Third Hospital, Beijing, China; b Department of Xiangya Medical Academic Promotion Center, Xiangya Hospital Central South University, Changsha City, China; c Department of General Surgery, Xiangya Hospital Central South University, Changsha City, China

**Keywords:** Triple-negative breast cancer, DRAIR, chemoresistance, recurrence

## Abstract

Diabetes regulated anti-inflammatory lncRNA (DRAIR) has been characterized as a critical player in type 2 diabetes mellitus. However, its role in other human diseases is unclear. Our preliminary sequencing analysis revealed an altered DRAIR level in triple-negative breast cancer (TNBC). We then explored the involvement of DRAIR in TNBC. In this study, plasma was collected from healthy controls (n = 60) and TNBC patients (n = 60). Non-tumor tissues and paired TNBC were also collected from TNBC patients. All TNBC patients received surgical resection of the primary tumors and chemotherapy. The 60 TNBC patients were divided into high and low plasma DRAIR level groups with median plasma DRAIR level as the cutoff value, and the occurrence of chemoresistance after treatment and tumor recurrence during a 5-year follow-up was monitored. Cell proliferation and viability were analyzed with BrdU assay and MTT assay, respectively. We found that plasma DRAIR levels were higher in TNBC patients than in controls. In addition, DRAIR expression in TNBC tissues was also significantly increased in TNBC tissues compared to the paired non-tumor tissues. Plasma DRAIR was positively and significantly related to DRAIR levels in TNBC tissues but not in non-tumor tissues. Patients in the high plasma DRAIR level group showed a significantly higher rate of chemoresistance after treatment and tumor recurrence during the follow-up. DRAIR promoted tumor cell proliferation and increased cell viability under doxorubicin treatment. Therefore, DRAIR is overexpressed in TNBC and predicts chemoresistance and tumor recurrence.

## Highlights

- DRAIR is overexpressed in TNBC;
- Plasma DRAIR is mainly from TNBC tissues;
- DRAIR promotes chemoresistance and tumor recurrence.

## Introduction

Breast cancer is the most commonly diagnosed malignant tumor among women in many countries worldwide [1,2]. It is estimated that more than 13% of women in the US will be diagnosed with breast cancer during their lifetime [3]. More than 60% of breast cancer patients are diagnosed at the localized stage or stage 1 [4]. With proper treatment, about 90% of patients with early-stage breast cancer can survive more than 5 years [4]. However, breast cancer has different subtypes with different prognoses. Triple-negative breast cancer (TNBC) is characterized by lacking the expression of estrogen, progesterone, and HER2, which are commonly detected in other types [5]. TNBC is not sensitive to hormone therapy and HER2 drugs. Thus, the prognosis of TNBC is generally poor [6,7].

The article "Diabetes regulated anti-inflammatory lncRNA is overexpressed in triple-negative breast cancer and predicts chemoresistance and tumor recurrence" was retracted in 2026. Reasons: concerns about the data; concerns about the results or conclusions.

Chemotherapy is the most frequently applied systemic treatment option for TNBC [8]. However, during the long-term use of chemical drugs, chemoresistance inevitably develops in many patients, leading to the failure of treatment [9]. Therefore, understanding the molecular mechanisms that mediate the resistance to chemical drugs in TNBC patients is the key to improving survival [9,10]. Long non-coding RNAs (LncRNAs) have no protein-coding capacity, but they regulate downstream gene expression to participate in cancer progression and the development of resistance to therapies [11–13]. Therefore, lncRNAs are potential targets to improve the treatment outcomes of chemotherapies [11–13]. However, the role of most lncRNAs in TNBC is unclear. Diabetes regulated anti-inflammatory lncRNA (DRAIR) has been characterized as a critical player in type 2 diabetes mellitus [14]. However, its role in other human diseases is unclear. Our preliminary sequencing analysis revealed an altered DRAIR expression level in TNBC (data not shown), indicating that DRAIR may also participate in TNBC. Therefore, we explored the involvement of DRAIR in TNBC, with a focus on its involvement in chemoresistance and tumor recurrence.

## Materials and methods

### Clinical samples

This study enrolled 60 TNBC patients and 60 healthy controls at Xiangya Hospital Central South University from May 2014 to May 2016. TNBC patients were diagnosed by immunohistochemistry. All patients received surgical resection of the primary tumors, and the tumors were dissected by experienced pathologists to prepare paired TNBC and non-tumor tissues. Blood was extracted from all TNBC patients and controls on the day of admission under fasting conditions to prepare plasma samples. All samples were stored in a liquid nitrogen tank. This study was approved by the Ethics Committee of this study (Supplemental file 1). All patients and controls signed informed consent. Table 1 shows the patients’ clinical data.

**Table 1.** Chi-squared analysis of the association between DRAIR expression in TNBC tissues and patients’ clinical data

Index	Number	DRAIR		P value
		Low (n = 30)	High (n = 30)	
Age				>0.05
≤60	28	15	13	
>60	32	15	17	
Histotype				>0.05
Ductal	52	25	27	
No ductal	8	5	3	
Tumor size				0.005
≤2 cm	18	14	4	
>2	42	16	26	
Lymph node metastasis				>0.05
Negative	36	20	16	
Positive	24	10	14	
Grade				>0.05
G1/G2	8	3	5	
G3	52	27	25	
Metastases				>0.05
Negative	42	20	22	
Positive	18	10	8	
Ki-67				>0.05
≤20%	10	6	4	
>20%	50	24	26	
Chemoresistance				0.03
Yes	20	6	14	
No	40	24	16	

The article "Diabetes regulated anti-inflammatory lncRNA is overexpressed in triple-negative breast cancer and predicts chemoresistance and tumor recurrence" was retracted in 2026. Reasons: concerns about the data; concerns about the results or conclusions.

### Treatment and follow-up

All 60 patients were treated with 4 cycles of full-dose doxorubicin (75 mg/m^2^ every 3 weeks). Tumor recurrence was monitored every month through the outpatient visit by biopsy and imaging analyses.

### Cells and transfections

Human TNBC cell lines MDA-MB-436 and SUM149PT from ATCC were cultured in DMEM medium (Cat # 11,054,001, Thermo Fisher Scientific, Shanghai, China) supplemented with 10% FBS (Cat # MFCD00132239, Sigma-Aldrich, Shanghai, China), streptomycin (10 μg/ml, Cat # 3810–74-0, Sigma-Aldrich, Shanghai, China) and penicillin (100 U/ml, Cat # 87–08-1, Sigma-Aldrich, Shanghai, China) in an incubator at 37°C with 95% humidity and 5% CO_2_.

MDA-MB-436 (ATCC, USA) and SUM149PT (ATCC, USA) cells were overexpressed with DRAIR by transfecting cells with DRAIR expression vector (pcDNA3.1) using Neon Electroporation Transfection device (Thermo Fisher Scientific, Shanghai, China). Transected cells were cultured in fresh media prior to subsequent assays.

### RNA isolation

Samples were first mixed with lysis buffer and kept at room temperature for 20 min prior to centrifugation. RNA samples were isolated using Quick-DNA/RNA™ Microprep Plus Kit (Cat # D7005, Zymo Research, Shanghai, China), and genomic DNA contamination was eliminated using DNase solution included in this kit. Nuclease-free water was used to elute RNA. After that, the concentration and integrity of RNA samples were analyzed using a Bioanalyzer. RNA concentration was adjusted to 1500 ng/μl. The integrity numbers of all RNA samples were higher than 8.5, indicating high RNA integrity.

### RT-qPCRs

cDNA samples were synthesized with about 1 μl RNA sample (1500 ng RNA) as the template through reverse transcriptions using ExcelRT™ Reverse Transcription Kit II (Smobio, Shanghai, China). About 1 μl cDNA samples were subjected to qPCRs on CFX96™ Real-Time PCR Detection System (Bio-Rad, Shanghai, China) to analyze DRAIR expression. Ct values were normalized to internal control 18S rRNA using the 2^–∆∆Ct^ method [15]. Primer sequences were 5’-GACTGTAGGCTGAAACTGA-3’ (forward) and 5’-TTCCGTGTCTTCGCTACT-3’ (reverse) for DRAIR and 5’-TAACCCGTTGAACCCCATT-3’(forward) and 5’-CCATCCAATCGGTAGTAG-3’ (reverse) for 18S rRNA.

### Cell proliferation (BrdU incorporation) assay [16]

Cells with satisfactory overexpression rates (> 4-fold) at 48 h post-transfection were harvested and washed with PBS. After about 3000 cells were seeded onto each well of a 96-well plate containing fresh medium mentioned above, cells were cultured for another 48 h and incubated with 10 μM BrdU (Cat # SAB4700630, Sigma-Aldrich, Shanghai, China) for 4 h. Cells incubated with the same volume of fresh media instead of BrdU were used as the blank control. Three replicate wells were set for each transfection group and control group. After that, cells were incubated with a peroxidase-coupled BrdU antibody (Sigma-Aldrich, Shanghai, China) for 2 h, and signals were developed by adding peroxidase substrate ethyl carbazole (Cat # 86–28-2, Sigma-Aldrich, Shanghai, China). OD values at 450 nm were measured to reflect cell proliferation and normalized to that of the control group, which was set to value ‘1’.

The article "Diabetes regulated anti-inflammatory lncRNA is overexpressed in triple-negative breast cancer and predicts chemoresistance and tumor recurrence" was retracted in 2026. Reasons: concerns about the data; concerns about the results or conclusions.

### MTT assay

Cells were collected using the methods described in BrdU incorporation assay and cultured in media containing 30 μM doxorubicin for 48 h. After incubated with 5 μl MTT solution (5 mg/ ml) for 2 h, cells in each well were incubated with 100 μl DMSO. OD values at 590 nm were measured to reflect cell viability and normalized to that of the control group, which was set to value ‘1’ [17].

### Statistical analysis

SPSS 22.0 software (IBM) was used for statistical analyses. Differences between two groups and among multiple groups were compared by Student’s t test and ANOVA Tukey’s test, respectively. Correlations were analyzed with Pearson’s correlation coefficient. The 60 TNBC patients were divided into high and low DRAIR level groups (n = 30). Associations between DRAIR expression and patients’ clinical data were analyzed by Chi-squared test. Recurrence-free curves were plotted and compared by log-rank test. Differences with a p-value smaller than 0.5 were considered statistically significant.

## Results

### Associations between DRAIR expression in TNBC tissues and patients’ clinical data

Association studies may provide insights into the functional analysis. To this end, the 60 TNBC patients were divided into high and low DRAIR level groups. Associations between DRAIR expression and patients’ clinical data were analyzed by Chi-squared test. It was observed that altered DRAIR level in TNBC tissues was closely correlated with tumor size and chemoresistance but not with age, histotypes, lymph node metastasis, tumor metastasis, grade, and Ki-67 (Table 1). Therefore, DRAIR may participate in tumor growth and the development of chemoresistance in TNBC.

### DRAIR expression pattern in TNBC

The altered expression suggests potential function. Therefore, total RNAs were extracted from paired TNBC and non-tumor tissues from 60 TNBC patients and subjected to RT-qPCRs to determine DRAIR expression. It was shown that DRAIR expression was significantly increased in TNBC tissues than in paired non-tumor tissues (Figure 1a, p<0.01, 2.43-fold). Differential DRAIR expression in plasma samples from 60 TNBC patients and 60 healthy controls were also analyzed by RT-qPCRs. It was observed that plasma DRAIR levels were higher in TNBC patients than in controls (Figure 1b, p<0.01, 2.52-fold).

The article "Diabetes regulated anti-inflammatory lncRNA is overexpressed in triple-negative breast cancer and predicts chemoresistance and tumor recurrence" was retracted in 2026. Reasons: concerns about the data; concerns about the results or conclusions.

**Figure 1.** DRAIR expression pattern in TNBC.

Total RNAs were extracted from paired TNBC and non-tumor tissues from 60 TNBC patients and subjected to RT-qPCRs to determine DRAIR expression (A). **, p < 0.01. Differential DRAIR expression in plasma samples from 60 TNBC patients and 60 healthy controls were analyzed by RT-qPCRs (B). **, p < 0.01.

### Correlations between DRAIR levels in tissue samples and plasma

To explore the potential source of plasma circulating DRAIR, Pearson’s correlation coefficient was applied to analyze the correlations between DRAIR expression in TNBC and non-tumor tissue samples and plasma DRAIR from 60 TNBC patients. Plasma DRAIR was significantly and positively related with DRAIR expression in TNBC tissues (Figure 2a, R^2^ = 0.8363, p < 0.0001) but not in non-tumor tissues (Figure 2b, R^2^ = 0.0452, p = 1027). Therefore, plasma DRAIR is mainly from TNBC tissues.

**Figure 2.** Correlations between DRAIR levels in tissue samples and plasma.

Correlations of plasma DRAIR with DRAIR expression in TNBC (A) and non-tumor (B) tissue samples from 60 TNBC patients were analyzed by Pearson’s correlation coefficient.

### Predictive value of plasma DRAIR for tumor recurrence

Tumor recurrence is correlated with poor survival. To explore the potential application of DRAIR in predicting tumor recurrence of TNBC patients, the 60 TNBC patients were divided into high and low plasma DRAIR level groups (n = 30). Their recurrence-free curves were plotted and compared by log-rank test. Compared to patients in low DRAIR level groups, patients in the high DRAIR level group experienced a significantly higher recurrence rate (Figure 3, p= 0.0147, hazard ratio = 3.007). Therefore, increased DRAIR expression may promote tumor recurrence in TNBC.

**Figure 3.** Predictive value of plasma DRAIR for tumor recurrence.

The 60 TNBC patients were divided into high and low plasma DRAIR level groups (n = 30), and their recurrence-free curves were plotted and compared by log-rank test.

### Role of DRAIR in the proliferation and viability of MDA-MB-436 and SUM149PT cells

Increased tumor cell proliferation and viability leads to tumor recurrence. To explore the role of DRAIR in TNBC cell proliferation, the proliferation of MDA-MB-436 and SUM149PT cells with DRAIR overexpressed was analyzed using BrdU assay. Compared to the controls, DRAIR overexpression significantly increased the proliferation of both cell lines (Figure 4a, p<0.01). Therefore, DRAIR may promote TNBC development and recurrence by promoting cancer cell proliferation. Moreover, the role of DRAIR in regulating TNBC cell viability under 30 μM doxorubicin treatment for 48 h was explored using MTT assay. We observed that DRAIR overexpression increased cell viability (Figure 4b, p<0.01), indicating that DRAIR might promote TNBC tumor recurrence by increasing tumor cell proliferation and viability.

The article "Diabetes regulated anti-inflammatory lncRNA is overexpressed in triple-negative breast cancer and predicts chemoresistance and tumor recurrence" was retracted in 2026. Reasons: concerns about the data; concerns about the results or conclusions.

**Figure 4.** Role of DRAIR in the proliferation of MDA-MB-436 and SUM149PT cells.

MDA-MB-436 and SUM149PT cells were overexpressed with DRAIR, and their proliferation was analyzed using BrdU assay (A). **, p < 0.01. MTT assay was conducted to explore the role of DRAIR in regulating TNBC cell viability under 30 μM doxorubicin treatment for 48 h (B). **, p < 0.01.

## Discussion

The present study explored the expression and function of DRAIR in TNBC. Our analysis revealed an increased DRAIR expression in both tumor tissues and plasma samples from TNBC patients. Moreover, DRAIR may participate in the chemoresistance and proliferation of TNBC cells.

The role of DRAIR has only been reported in monocytes collected from patients with type 2 diabetes mellitus, in which DRAIR is under-expressed [14]. It was observed that DRAIR negatively regulates inflammatory responses in monocytes of a diabetic animal model by interacting with chromatin and suppressing H3K9me2 and G9a expression [14]. Based on our knowledge, the role of DRAIR in other human diseases is unclear. The present study reported an increased DRAIR expression in both plasma and tumor tissues of TNBC patients. Interestingly, plasma DRAIR is only positively correlated with DRAIR in TNBC tissues but not in non-tumor tissues. Therefore, TNBC tissues are likely the main source of circulating DRAIR in plasma. DRAIR may participate in TNBC mainly by accelerating tumor cell proliferation. This speculation is supported by the observation that DRAIR is closely correlated with tumor size but not tumor metastasis. In addition, DRAIR overexpression increases TNBC cell proliferation.

The development of chemoresistance is common in TNBC patients [18]. The present study showed that increased DRAIR expression is closely associated with the development of chemoresistance in TNBC patients. Therefore, measuring DRAIR expression level prior to treatment may predict chemoresistance, thereby improving treatment outcomes by redesigning treatment strategies. This study also revealed that the recurrence of TNBC after treatment is closely related to plasma DRAIR in TNBC patients. Together with the observation of the enhancing effects of DRAIR on TNBC cell proliferation, we speculated that DRAIR could increase TNBC cell proliferation to promote recurrence. Therefore, DRAIR inhibition may serve as a potential target to suppress TNBC recurrence. However, *in vivo* experiments are needed to test our hypothesis.

The article "Diabetes regulated anti-inflammatory lncRNA is overexpressed in triple-negative breast cancer and predicts chemoresistance and tumor recurrence" was retracted in 2026. Reasons: concerns about the data; concerns about the results or conclusions.

The function of lncRNAs in TNBC has been explored previously [19]. Moreover, the role of lncRNAs in the development of chemoresistance in multiple cancers has also been extensively studied [20,21]. However, the role of lncRNA in TNBC recurrence is hardly known. Our study reported a novel biomarker for tumor recurrence in TNBC.

## Conclusion

DRAIR is overexpressed in both tumor tissues and plasma samples from TNBC patients and may participate in chemoresistance and proliferation of TNBC cells.

## Data Availability

The datasets generated during and/or analyzed during the current study are not publicly available but are available from the corresponding author on reasonable request.

## List of Abbreviations

TNBC: triple-negative breast cancer
